# Development and Maturation of the Immune System in Preterm Neonates: Results from a Whole Genome Expression Study

**DOI:** 10.1155/2014/498318

**Published:** 2014-05-28

**Authors:** Magdalena Zasada, Przemko Kwinta, Wojciech Durlak, Mirosław Bik-Multanowski, Anna Madetko-Talowska, Jacek Józef Pietrzyk

**Affiliations:** ^1^Department of Pediatrics, Polish-American Children's Hospital, Faculty of Medicine, Jagiellonian University, Wielicka 265, 30-663 Krakow, Poland; ^2^Department of Medical Genetics, Polish-American Children's Hospital, Faculty of Medicine, Jagiellonian University, Krakow, Poland

## Abstract

To expand the knowledge about the consecutive expression of genes involved in the immune system development in preterm neonates and to verify if the environment changes the gene expression after birth we conducted a prospective study that included three cohorts: (A) extremely (gestational age (GA): 23–26 weeks; *n* = 41), (B) very (GA: 27–29 weeks; *n* = 39), and (C) moderately preterm infants (GA: 30–32 weeks; *n* = 33). Blood samples were drawn from the study participants on the 5th and 28th day of life (DOL). The mRNA samples were evaluated for gene expression with the use of GeneChip Human Gene 1.0ST microarrays. Differential expression analysis revealed small subsets of genes that presented positive or negative monotone trends in both the 5th (138 genes) and 28th DOL (308 genes) in the three subgroups of patients. Based on pathway enrichment analysis, we found that most of the pathways that revealed a positive monotone trend were involved in host immunity. The most significantly GA dependent pathways were T-cell receptor signaling pathway and intestinal immune network for IgA production. Overall 4431 genes were differentially expressed between the 5th and 28th DOL. Despite differences in gestational age, patients with the same postconceptional age have a very similar expression of genes.

## 1. Introduction

According to the current statistics, invasive neonatal infections are responsible for about 36% of the estimated 4 million neonatal deaths annually [1]. Survivors of neonatal sepsis have an increased risk of prolonged hospital stay, adverse neurodevelopmental sequelae, and bronchopulmonary dysplasia [2, 3]. The prevalence of neonatal sepsis is inversely correlated with gestational age and birth weight; therefore, infants born prematurely are particularly highly prone to developing infection [4]. One of the major causes of increased incidence of sepsis in premature neonates is the immaturity of their immune system [5].

The development of the fetal immune system begins at 4.5–6 weeks of gestation. Throughout gestation two major systems of fetus defense gradually develop: the nonspecific innate immune mechanism and the adaptive immune system [6]. Mechanisms of innate immunity operate effectively without prior exposure to a microorganism or its antigens.

Adaptive immune response is relatively immature at birth due to limitations of exposure to antigens in utero and due to the impaired functions of B and T cells. Therefore, the protection of the neonate against infection mainly depends upon passively acquired antibodies transferred from the mother and components of the innate immune system [7].

The ontogenesis of the immune system correlates with the developmental age of the fetus, but little is known when each of the respective aspects of the immune system matures normally in utero and what the consequences of the premature birth on these processes are.

It is known from studies conducted so far that the premature neonates show both qualitative and quantitative deficits in comparison with an adult or term neonate immune response. These studies were based on quantitative evaluation of the elements (cells, receptors) [8] of the immune system or comparison of their function. There are also studies evaluating the expression of individual genes involved in the development of the immune system in infants with variable degrees of prematurity [9].

The introduction of the microarray technique into clinical studies was one of the most important turning points responsible for the dramatic progress in the field of human genetics during the last decade.

The aim of the study was to evaluate the consecutive expressions of genes involved in the immune system development in preterm neonates and to verify if the environment changes the gene expression after birth.

## 2. Methods

A prospective study was conducted between September 1, 2008, and November 30, 2010. The entry criteria were (a) preterm birth <32 weeks gestational age, (b) birth weight ≤1500 g, and (c) the need for respiratory support. All patients were outborn in local hospitals and transported to the Polish-American Children's Hospital, which is a tertiary care unit for the region.

The majority of patients are referred from first-level neonatal care hospitals, which provide mainly for rural areas. Detailed perinatal history (birth weight, gestational age, and Apgar score at 1 and 5 minutes after birth) and history of treatment in the referral hospital (mechanical ventilation, oxygen therapy, surfactant treatment, and diagnoses) were taken on admission. Maternal fever/infection was used as surrogate for “clinical diagnosis of chorioamnionitis.” Data on histological chorioamnionitis were unavailable in most cases. Ureaplasma infection was defined as positive tracheal aspirate culture for* Ureaplasma urealythicum*. The study was approved by the Ethics Committee of the Jagiellonian University, Faculty of Medicine (KBET 27/B/2007). Written informed consent was obtained from the parents of all participants involved in the study.

### 2.1. Characteristics of the Studied Group

One hundred and twenty newborns were included in the study. The mean birth weight was 1029 g (SD: 290), and the mean gestational age was 27.8 weeks (SD: 2.5). The majority of the pregnancies were terminated by abrupt deliveries. Seven newborns died before the end of the first month of life; therefore, 113 children were included in the final analysis.

Forty-one infants were included in the extremely preterm cohort, 39 infants in the very preterm cohort, and 33 infants in the moderately preterm cohort. The clinical characteristics of the studied cohorts were presented in Table 1.

### 2.2. Microarray Analysis

After obtaining written informed consent from the parents, blood samples (0.3 mL) were drawn from all the study participants on the 5th and 28th day of life (DOL) for the assessment of whole genome expression in peripheral blood leukocytes. Subsequently, Ficoll isopaque gradient centrifugation (30 min, 2100 rpm, RT), two times wash in 1x PBS (12 min, 1600 rpm, 40°C), and finally RiboPure Blood Kit (Ambion, Life Technologies, Carlsbad, USA) were used for total RNA extraction. RNA concentration was measured with the use of NanoDrop Spectrophotometer (NanoDrop ND-1000; Thermoscientific, Waltham, USA), and RNA quality was determined by 2100 Bioanalyzer (Agilent, Santa Clara, USA).

100 ng of total RNA was used for the single microarray experiment. GeneChip Human Gene 1.0 ST Arrays (Affymetrix, Santa Clara, USA) were used. Whole transcript microarray experiment was performed. Details of microarray experiment were published previously [10].

### 2.3. Real-Time PCR Validation

To validate the results obtained by the microarray analysis real-time PCR technique was used. A total of 30 cDNA samples remaining after microarray analysis (30 patients) were used for the validation procedure. Samples were randomly selected from the studied groups.

From each sample 100 ng of cDNA was used for the single TaqMan Gene Expression Assay, and the expression level of 14 randomly selected genes was determined. Amplification reaction was performed with the use of TaqMan Universal PCR Master Mix and appropriate TaqMan probes (Life Technologies, Carlsbad, USA). Each sample was analyzed in duplicate.

Average between the expressions of endogenous controls (housekeeping genes: GAPDH and Actin-B) was used for determination of the relative expression levels with the use of ΔΔCt calculation.

Following TaqMan Gene Expression Assays were used: Hs00900055_m1 (VEGF gene), Hs00952786_m1 (AK5 gene), Hs00217864_m1 (OLAH gene), Hs01030384_m1 (ILR2 gene), Hs00187022_m1 (ADAM23 gene), Hs00736937_m1 (DAAM2 gene), Hs00360669_m1 (CD177 gene), Hs00255338_m1 (KLRC4 gene), Hs00171191_m1 (FBN1 gene), Hs00539582_s1 (LRRN3 gene), Hs00196254_m1 (NELL2 gene), Hs00924296_m1 (MPO gene), Hs00541549_m1 (ABCA13 gene), Hs00197437_m1 (OLFM4 gene), GAPDH (Hs02758991_g1), and Actin-B (Hs99999903_m1) (Life Technologies, Carlsbad, USA).

### 2.4. Predefined Comparisons

Based on gestational age the studied group was divided into three cohorts: (a) extremely preterm infants (born below 27 weeks of gestation), (b) very preterm infants (born between 27 and 29 weeks of gestation), and (c) moderately preterm infants—born between 30 and 32 weeks of gestation. Gene expression profile was compared between the cohorts on the 5th and 28th DOL. Moreover, the changes between expression values between 5th and 28th DOL of whole study group were analyzed, too. The final step of analysis included comparison between the results of gene expression recorded on the 28th DOL in the group of extremely preterm infants and the results of gene expression recorded on the 5th DOL in the group of very preterm infants. The last comparison provided opportunity to compare both groups in the similar postmenstrual age.

### 2.5. Statistical Analysis

Basic demographic data were compared using the one-way analysis of variance or Kruskal-Wallis analysis of variance as appropriate. Qualitative values were compared using the chi-square test.

Neonatal data used for the study was recorded daily during hospitalization in NICU in a prospective manner and stored in computer databases. For the purpose of the study the following data was used: sex, birth weight, gestational age, intrauterine growth parameters, Apgar score, incidence of preeclampsia, maternal diabetes, preterm rupture of membranes, chorioamnionitis, delivery type, delivery room management, presence of respiratory distress syndrome (RDS), length of mechanical ventilation, surfactant administration, use of ibuprofen for patent ductus arteriosus (PDA), PDA ligation, early- and late-onset septic episodes, ureaplasma infection, prevalence of intraventricular hemorrhage (IVH), periventricular leukomalacia (PVL), weight gain during NICU stay, and length of hospitalization. The microarray data were preprocessed using the R/Bioconductor package aroma.affymetrix [11, 12]. For normalization we used robust multiarray average (RMA) [13]. Quality control was performed by investigating* principal component analysis *(PCA),* relative log expression* (RLE), and* normalized unscaled standard error *(NUSE) plots. None of the arrays were discarded due to poor quality [14].

Moderated* t*-tests were performed to detect the probes that were differentially expressed between groups, using the* limma* package in the R statistical software [15]. For the three categories of gestational age we used Spearman's rho statistic to test whether there was a monotonic trend in gene expression between the categories [16].

Multiple testing corrections, using the Benjamini-Hochberg procedure, were applied to control the false discovery rate (FDR) [17]. If a probe set had a corrected for multiple comparison *P* value less than 0.01, it was declared significantly differentially expressed.

DAVID annotation tools were used to explore which predefined gene sets were significantly enriched in one group compared to another [18]. The KEGG (*Kyoto Encyclopedia of Genes and Genomes*; http://www.genome.jp/kegg/) pathways were selected for analysis. Genes differentially expressed between the groups with *P* values adjusted for multiple testing below 0.01 were used as input for pathway enrichment analysis in DAVID.

The mean fold change values representing differences in expression between the groups with regard to each of the 14 genes selected for validation were compared between the microarray and the TaqMan Gene Expression experiments. Student's* t*-test was used for evaluating the statistical significance of observed differences between gene expressions.

All data were collected and analyzed in the adherence to the Minimal Information about a Microarray Experiment guidelines. All primary microarray data were submitted to GEO public repository and are accessible through GEO Series accession number GSE32472 (http://www.ncbi.nlm.nih.gov/geo/query/acc.cgi?acc=GSE32472).

## 3. Results

### 3.1. Whole Genome Expression

One hundred and thirty-eight genes presented a monotone trend on the 5th and 308 on the 28th day of life. A summary of the number of differentially expressed genes between the groups is presented in Table 2.

4431 genes were differentially expressed between 5th and 28th DOL (paired* t*-test), including 1522 genes whose expression increased with time and 2909 genes whose expression decreased with time. The difference in expression measured as a fold change ranged between 1.0 and 1.5 in the majority of genes. Only 487 genes have shown the difference in expression greater than 1.5.

When the samples collected on 28th DOL in extremely preterm infants and on 5th DOL in very preterm infants were compared, the expressions of 176 genes were significantly higher in the group of extremely preterm infants and the expressions of 186 gene genes were significantly lower. The difference in expression measured as a fold change of 56 genes was greater than 1.5.

### 3.2. Pathway Enrichment Analysis

Differentially expressed genes (with *P* values adjusted for multiple testing below 0.01) were used as input for pathway enrichment analysis in DAVID.

A summary of the analysis is presented in Table 3. There was no pathway upregulated in the group of extremely preterm infants neither on the 5th DOL nor 28th DOL. However, 4 pathways were downregulated on 5th DOL and 5 pathways were downregulated on 28th DOL in the group of extremely preterm infants. Among above-mentioned pathways, three were downregulated in both time points: T-cell receptor signaling, hematopoietic cell lineage, and intestinal immune network for IgA production pathways.

The differentially expressed genes between 5th and 28th DOL studies belonged to 21 pathways; 12 pathways were upregulated and 9 pathways were downregulated. Among 12 pathways whose expression was higher on 28th DOL than on 5th DOL were T-cell receptor signaling, hematopoietic cell lineage, and intestinal immune network for IgA production pathways.

When the expression of genes on the 28th DOL in the group of extremely preterm infants was compared to expression on the 5th DOL in the group of very preterm infants, only 3 pathways were differentially upregulated. Surprisingly, there was no pathway downregulated.

### 3.3. Real-Time PCR Validation

The validation procedure did not reveal significant differences between the results obtained with use of microarrays compared to real-time PCR technique [10].

## 4. Discussion

The use of microarrays has provided a new opportunity for studying even 20000 human genes in a single experiment. The greatest advantage of this method is that it enables the assessment of a huge number of genetic factors (practically all human gene expression), while only a small amount of blood is necessary for testing, which is very important in preterm neonates.

In this study we assessed the whole genome expression in a cohort of preterm neonates in the 5th and 28th day of life. The cohort was subdivided into three groups depending on the gestational age (extremely preterm, very preterm, and moderately preterm), as described above. The genomic expression was compared between these three groups. To our knowledge this cohort is the first one designed to assess the whole genome expression among preterm neonates. The nature of the study was mainly exploratory.

Differential expression analysis revealed small subsets of genes that presented positive or negative monotone trends in both the 5th and 28th DOL in the three subgroups of patients, depending on the gestational age. On the contrary, we found a much higher number of genes that revealed positive or negative monotone trends when we compared gene expression between the 5th and 28th DOL in the whole cohort. In this comparison, significantly more genes were underexpressed in the 28th DOL rather than overexpressed. Finally we attempted to assess the impact of the extrauterine environment on genomic expression and compared the group of extremely preterm newborns on 28th DOL with very preterm newborns on 5th DOL. The analysis revealed a comparable number of genes that were over- and underexpressed.

Using pathway enrichment analysis, which allows us to identify network expression alterations that may be insignificant on the level of individual genes, we identified pathways that were differentially regulated with regard to gestational age. We found that most of the pathways that revealed a positive monotone trend on both the 5th and 28th DOL between all three age groups are involved in host immunity. Similarly we observed a significantly higher expression of pathways involved in immune response when we compared patients on 5th and 28th DOL, regardless of the gestational age. Both analyses revealed a relative increase in T-cell receptor signaling pathway and intestinal immune network for IgA production.

### 4.1. T-Cell Receptor Signaling Pathway

The neonatal immune system, both innate and adaptive, bears features of functional immaturity and therefore significantly contributes to neonatal morbidity and mortality [6, 19, 20]. The innate immune system is the first line of defense against invading pathogens that include numerous mechanisms such as skin and mucosal barriers, cellular network (neutrophils, monocytes, antigen-presenting cells, and natural killer cells), toll-like receptors (TLR), and humoral factors (e.g., complement). It can operate sufficiently without previous exposure to antigens in term newborns, and due to the limited fetal exposure to antigens it is a major protective mechanism for the newborn [6, 21]. The major innate immune system involves TLRs, which are dedicated to recognize PAMP (pathogen associated molecular pattern). However, it has been shown that the innate immune system reveals features of immaturity in prematurely born newborns. Recent study by Tissières et al. [5] proves that the level of cytokines involved in innate immune response is lower in preterm than in term newborns and, interestingly, that this deficiency could be reversed by treatment with interferon-*γ*.

Conversely, the adaptive immune response requires antigen exposure and develops gradually after birth. In newborns, cytokine production in response to stimuli exhibits polarization with Th-1 response downregulation [22, 23]. Th-1 cytokine production impairment has been presupposed to be involved in decreased defensive mechanisms against viral pathogens, including HSV [24], CMV [25], and other intracellular pathogens like* Listeria spp.*,* Toxoplasma* [26], or* Mycobacterium tuberculosis*, particularly in preterm newborns.

In the current study we demonstrated for the first time a coherent trend of increasing expression of genes involved in T-cell receptor signaling with increasing gestational and chronological age. The functional changes of the developing immune system, including regulatory T-cell (Treg) maturation [27], monocyte stimulation ability [28], complement system [29], or T-cell response to Toll-like receptor ligands (for example, LPS) [30], have been described in previously published papers. Our results might reflect dynamic maturational changes involved in the development of fetal adaptive immunity mechanisms that could be responsible for the increased risk of serious infections and mortality in extremely premature newborns.

### 4.2. Intestinal Immune Network for IgA Production

Intestinal immunity consists of two major components—innate defenses (gastric acid, protolithic enzymes, intestinal mucin, permeability, defensins, cathelicydins, and lectins (REG3_*γ*_) [31] and active immunity (T and B lymphocytes, secretory IgA). After induction of mucosal B cells in the Peyer's patches, B cells circulate through the bloodstream to the mesenteric lymph node and enter the intestinal submucosa, where they start to produce IgA, which is subsequently exported by means of transcytosis across the intestinal membranes [32]. IgA protects against bacterial, parasitic, and viral mucosal pathogens by neutralizing toxins and blocking the adherence and penetration of microorganisms. It can also induce effector immune responses and therefore maintain the intestinal microflora and immune homeostasis [33–35]. In our study we demonstrated that the expression of genes from the intestinal immune network for IgA production increases with postconceptional age. This fact may be connected with gradually increasing host defenses in premature babies against toxins and microorganisms.

Apart from genetic predisposition, disruption of the intestinal barrier secondary to hypoxic mucosal injury, bacterial colonization and formula feeding, immaturity of the gut mucosal immunity, and a relative deficiency of sIgA in the premature neonate have been implicated as a potential risk factor for NEC [36, 37]. Secretory IgA (sIgA) has been recognized as a critically important component of mucosal defence and some of the protective effects of human colostrum and milk against NEC have been attributed to its sIgA content [36]. According to Anderson and Kliegman [38], supplementation of enteral immunoglobulin rich in IgA can reduce the risk of NEC. We can speculate that the increasing gene expression of the intestinal immune network for IgA production pathway may be connected with diminishing the risk of developing NEC in maturing preterm neonates.

We know that birth initiates the conversion from the intrauterine sterile environment to the extrauterine confrontation with microbial and food antigens. This stimulus has a profound effect on the maturation of mucosa associated lymphatic tissues (e.g., Peyer's patches) and other lymphoid tissues [39, 40]. But surprisingly, despite the massive exposure to foreign antigens (dietary antigens-formula milk or breast milk and skin-to-skin contact), enabling the colonization with commensals earlier than in neonates from group B, the gene expression of the intestinal immune network for IgA production did not differ between the youngest preterm babies from group A in their 28th DOL and children from group B in their 5th DOL (when they reached the same postconceptional age). It is possible that maturational steps involved in the ontogenesis of the intestine immune system are genetically regulated and antigen exposure does not trigger any acceleration in their development (they are independent from the extrinsic factors). Similar results were obtained by Rogosch et al. [41], who confirmed that preterm birth did not measurably accelerate the maturation of the IgA repertoire.

## 5. Limitations of the Study

Our studied groups varied significantly with the percentage of children whose mothers received antenatal steroids. According to the literature, prenatal use of steroids may influence gene expression in children born preterm [42]. In our population the rate of prenatal steroid was low, so it is possible that in other populations where the usage of prenatal steroids is higher, the results may be different.

The effect of congenital infection, which was present in some of our patients, may influence gene expression.

All children included in our study were transferred from regional hospitals and the aim of the study was to assess the role of environmental factors occurring after birth. It should be noted that it was not feasible to directly assess the potential role of intrauterine factors, for example, by means of analysis of pattern of genome expression in lymphocytes obtained from cord blood samples. This situation might bias our results. Unfortunately, even assessment of cord blood samples would reflect only the very last phase of pregnancy, directly preceding the preterm delivery, which was triggered by various factors and not the physiological phenomena during pregnancy.

Last but not least, it should be noted that this investigation was performed in leukocytes, not, for example, in intestine tissues, which raises the question of whether gene expression of white blood cells reflects gene expression in the peripheral tissue. However, according to some researches, around 90% of transcripts are coexpressed in different tissues of the body, for example, in peripheral blood mononuclear cells and skeletal muscle cells [43].

## 6. Conclusion

Based on pathway enrichment analysis, we identified a few pathways which presented a positive monotone trend during the gestational age; most of them are involved in host immunity. We were not able to identify any pathway where expression of genes decreases with the gestational age. Despite differences in gestational age, patients with the same postconceptional age have a very similar expression of genes. The results are of sufficient interest to warrant further investigation on this subject.

## Figures and Tables

**Table 1:** Comparison of selected demographic data in the studied cohorts.

	Extremely preterm (23–26 weeks) (*n* = 41)	Very preterm (27–29 weeks) (*n* = 39)	Moderately preterm (30–32 weeks) (*n* = 33)	*P*
Birth weight, g (*x* ± SD)	727 ± 124	1149 ± 207	1245 ± 211	<0.001^a^
Gestational age (weeks) (*x* ± SD)	25.0 ± 1.1	28.2 ± 0.8	30.7 ± 0.8	<0.001^a^
Male gender	24 (58%)	20 (51%)	17 (52%)	0.76^b^
Vaginal delivery/Cesarean section	20/21	15/24	8/25	0.01^b^
Multiple pregnancy	4 (10%)	8 (20%)	6 (18%)	0.56^b^
Small-for-gestational-age infant	4 (10%)	1 (2%)	5 (15%)	0.1^b^
Maternal hypertension	8 (19%)	7 (18%)	2 (8%)	0.74^b^
Maternal diabetes	3 (7%)	2 (5%)	0	0.79^b^
Maternal fever/infection prior to delivery	5 (12%)	6 (15%)	4 (13%)	0.8^b^
1st minute Apgar score (Me; 25–75th percentile)	2 (1–4)	5 (4–6)	5 (2–6)	0.01^c^
5th minute Apgar score (Me; 25–75th percentile)	6 (4–6)	7 (6-7)	7 (6–8)	0.001^c^
Delivery room intubation	28 (69%)	16 (40%)	11 (33%)	0.01^b^
Surfactant therapy	33 (81%)	29 (73%)	14 (43%)	0.003^b^
Initial a/A ratio	0.31 ± 0.2	0.25 ± 0.13	0.44 ± 0.25	0.01^a^
Prenatal steroids	10 (25%)	12 (29%)	22 (66%)	0.01^b^
Ureaplasma infection	12 (29%)	8 (21%)	6 (18%)	0.28^b^
Pharmacological closure of patent ductus arteriosus	22 (54%)	23 (59%)	11 (33%)	0.08^b^
Surgical closure of patent ductus arteriosus	18 (44%)	4 (10%)	2 (6%)	<0.001^b^
Length of mechanical ventilation (Me; 25–75th percentile)	42 (25–52)	3 (1–10)	2 (0–6)	<0.001^c^
Bronchopulmonary dysplasia	40 (98%)	24 (62%)	6 (18%)	<0.001^b^

^a^ *P* value for one-way analysis of variance.

^b^ *P* value for chi-square test.

^c^ *P* value for Kruskal-Wallis analysis of variance.

**Table 2:** Summary of the number of differentially expressed genes between the studied groups.

Comparison		*P* < 0.01 adjusted for multiple comparison *P* < 0.01	*P* < 0.01; fold change >1.5
5th DOL	Genes presented a positive monotone trend (expression in extremely preterm is lower than that in very preterm; expression in very preterm is lower than that in moderately preterm)	56	
	Genes presented a negative monotone trend	82	

28th DOL	Genes presented a positive monotone trend	253	
	Genes presented a negative monotone trend	55	

5th DOL versus 28th DOL (paired *t*-test)	Genes whose expressions were significantly higher on the 28th DOL compared to those on the 5th DOL	1522	150
	Genes whose expressions were significantly lower on the 28th DOL compared to those on the 5th DOL	2909	337

Extremely preterm infants measurement on the 28th DOL versus very preterm infants measurements on the 5th DOL	Genes whose expressions were significantly higher in the group of extremely preterm infants compared to those in the group of very preterm infants	176	29
	Genes whose expressions were significantly lower in the group of extremely preterm infants compared to those in the group of very preterm infants	186	27

**Table 3:** Summary of the pathway analysis for the differentially expressed genes between the groups. Pathways with FDR value less than 15% are shown.

Input to pathway analysis	Pathway name	FDR (%)
Genes presented a positive monotone trend on the 5th DOL, adjusted for multiple comparison *P* < 0.01 (expression in extremely preterm is lower than that in very preterm; expression in very preterm is lower than that in moderately preterm)	T-cell receptor signaling pathway Cell adhesion molecules (CAMs) Hematopoietic cell lineage Intestinal immune network for IgA production	0.6 1.3 3.7 12.5

Genes presented a negative monotone trend on the 5th DOL, adjusted for multiple comparison *P* < 0.01	No pathway	

Genes presented a positive monotone trend on the 28th DOL, adjusted for multiple comparison *P* < 0.01	Primary immunodeficiency T-cell receptor signaling pathway Hematopoietic cell lineage Intestinal immune network for IgA production Cytokine-cytokine receptor interaction	0.01 0.02 1.3 4.9 10.5

Genes presented a negative monotone trend on the 28th DOL, adjusted for multiple comparison *P* < 0.01	No pathway	

Genes whose expressions were significantly higher on the 28th DOL compared to those on the 5th DOL (paired *t*-test, *P* < 0.01; fold change > 1.5)	Graft-versus-host disease Allograft rejection Antigen processing and presentation Intestinal immune network for IgA production Cell adhesion molecules (CAMs) Primary immunodeficiency Hematopoietic cell lineage Natural killer cell-mediated cytotoxicity Cytokine-cytokine receptor interaction B-cell receptor signaling pathway T-cell receptor signaling pathway Jak-STAT signaling pathway	<0.001 <0.001 <0.001 <0.001 <0.001 0.03 0.04 0.13 0.5 1.8 5.8 6.0

Genes whose expressions were significantly lower on the 28th DOL compared to those on the 5th DOL (paired *t*-test, *P* < 0.01; fold change > 1.5)	Cell cycle Regulation of actin cytoskeleton Fc gamma R-mediated phagocytosis Glycolysis/gluconeogenesis Lysosome Endocytosis Base excision repair Leukocyte transendothelial migration Glutathione metabolism	0.27 1.04 1.09 1.54 3.46 3.50 5.69 7.59 8.30

Genes whose expressions were significantly higher in the group of extremely preterm infants (measurements on the 28th DOL) compared to those in the group of very preterm infants (measurements on the 5th DOL); *P* values adjusted for multiple testing, *P* < 0.01	Graft-versus-host disease Cytokine-cytokine receptor interaction Natural killer cell-mediated cytotoxicity	0.01 0.4 2.3

Genes whose expressions were significantly lower in the group of extremely preterm infants (measurements on the 28th DOL) compared to those in the group of very preterm infants (measurements on the 5th DOL); *P* values adjusted for multiple testing, *P* < 0.01	No pathway	
